The article "Evaluation of the Emotion Model in Electronic Music Based on PSO-BP" was published in 2022. Journal: Comput Intell Neurosci.

# Evaluation of the Emotion Model in Electronic Music Based on PSO-BP

**DOI:** 10.1155/2022/5601689

**Published:** 2022-05-30

**Authors:** Ting Guo

**Affiliations:** School of Music, Xi'an University, Xi'an, Shannxi 710065, China

## Abstract

Electronic music can help people alleviate the pressure in life and work. It is a way to express people's emotional needs. With the increase of the types and quantity of electronic music, the traditional electronic music classification and emotional analysis cannot meet people's more and more detailed emotional needs. Therefore, this study proposes the emotion analysis of electronic music based on the PSO-BP neural network and data analysis, optimizes the BP neural network through the PSO algorithm, and extracts and analyzes the emotional characteristics of electronic music combined with data analysis. The experimental results show that compared with BP neural network, PSO-BP neural network has a faster convergence speed and better optimal individual fitness value and can provide more stable operating conditions for later training and testing. The electronic music emotion analysis model based on PSO-BP neural network can reduce the error rate of electronic music lyrics text emotion classification and identify and analyze electronic music emotion with high accuracy, which is closer to the actual results and meets the expected requirements.

## 1. Introduction

With the popularity of the Internet and mobile communication devices, music, as a value-added service of Internet and mobile devices, has developed rapidly in recent years. The study of music emotion recognition is an important technical link in music operation and maintenance service. There are two research directions in the field of music emotion recognition: one direction is to extract the tone feature value by wavelet transform and recognize the related tones. This kind of music file stores the sampling data of music acoustic signal. The research focuses on signal processing. The other direction is to use HMM (hidden Markov model) for single tone note recognition, that is, to use the audio signal of music to obtain the score reflecting the music content. Due to the heavy workload of identifying each note in music, it is impossible to accurately identify the emotional type of music. The existing music emotion classification methods have the following two shortcomings: (1) the tone recognition method is based on the sampling data processing of music acoustic signal, unable to recognize music emotion information. (2) Analyze music emotion based on the pitch, length, and intensity of a single note. BP neural network has been successful in many fields because it can correct the weight and threshold according to the backpropagation of error. However, it may fall into local minima and cannot ensure convergence to the global minima. In addition, the number of backpropagation training is large and the convergence speed is slow, which makes the learning results sometimes unsatisfactory. If the particle swarm optimization algorithm with the mean square error index as the fitness value is used to train the weight of BP network, it will get a faster convergence speed and avoid the occurrence of the local maximum.

Music plays a very important role in people's life, work, and study. Music can not only help people reduce the pressure in life and work but also express rich emotions and affect people's mood and heart. It is an indispensable part of the development of human society. With the changes of the times, the way people listen to music has changed from tape records to digital music files, and the types of music are also increasing. With the continuous development of the Internet and technology, electronic music has gradually entered the public's vision and occupied a certain position in the music market. Different people have different preferences for different electronic music, and if people want to obtain their preferred electronic music types, they have to choose from a large number of electronic music, which greatly increases the time cost of listening to music [1]. Therefore, how to quickly and accurately select and listen to much needed electronic music has become the focus of electronic music classification research. Music emotion analysis and recognition are the key basis to improving the classification and search efficiency of electronic music. In the past, electronic music recognition mainly used wavelet transform to extract the characteristics of musical tones and then identify and analyze them or recognize the single tone notes of music through music audio signals [2]. The former method cannot identify the emotional information in electronic music, while the latter method is inaccurate. Neither method can meet people's needs for emotional analysis of electronic music.

The development of artificial intelligence and data analysis technology opens up a new development direction for electronic music emotion analysis. Therefore, this paper proposes electronic music emotion analysis based on the PSO-BP neural network and data analysis, which is optimized by the PSO algorithm on the basis of the BP neural network structure to improve the performance of the neural network. At the same time, combined with data analysis, the music emotion characteristics of electronic music are extracted and processed through the music emotion analysis model so as to obtain the expected analysis of electronic music emotion. This paper is mainly divided into three parts. The first part is the development of music emotion classification and analysis and related research. The second part is the construction of electronic music emotion analysis model based on PSO-BP neural network. The fourth part is the application experiment and result analysis of the electronic music emotion analysis model based on the PSO-BP neural network.

## 2. Related Work

Music emotion analysis is closely related to the development of artificial intelligence. People put forward the idea of recognizing the emotion expressed by music based on this and combined it with corresponding computer technology in the early stage of the development of artificial intelligence so that artificial intelligence can realize the functions of music, self-action music, and emotional music retrieval [3]. There are some similarities between music emotion classification and analysis research and speech emotion analysis, and the biggest difference between the two is that the duration of music is longer, and the content composition is more complex. If emotion analysis needs to extract a large number of emotional features from music, it has many dimensions and has high difficulty in feature analysis [4]. The key influencing factors of music emotion analysis results are characteristic parameters and classification methods, which is also an important research direction for most scholars.

In foreign countries, the research on music emotion analysis has achieved good results and has begun to be applied. For example, Japan's “chuyin” software converts the input tone and lyrics into sound and converts the songs accordingly through emotional parameters so as to obtain music works comparable to real-life performance [5]. In addition, some scholars pointed out that music style can classify music emotion with the help of chord and beat information in music, but such music emotion classification method has certain limitations in the fine-grained aspect of emotion classification [6]. Other scholars extracted Mel frequency based on the frequency domain, combined with a genetic classification algorithm, and classified music emotion information with spacing and zero-crossing rate as the best fitting ratio, and achieved good results [7]. With the increase of music emotion classification and analysis methods, some scholars have studied the performance of different modal features in two-dimensional emotion coordinates. The research results show that compared with lyrics text classification, the effect of the deep learning method in audio classification results is better [8]. In music, the emotional classification of lyrics text is also an important part. Its classification technology comes from the text classification model. That is, the computer extracts the corresponding features of the formulated documents and automatically assigns them to the categories defined according to the text content [9]. Text classification mainly includes two parts: text feature extraction and classification. On this basis, some scholars have proposed a lyric emotion classification method. That is, the emotional features of lyrics are extracted through partial syntactic analysis and then classified and verified by naive Bayes and machine learning methods [10]. With the development of a deep learning algorithm, some scholars classify Indonesian songs and lyrics into happy and sad music emotions through the recurrent neural network, and its highest accuracy can reach 82% [11].

The research on the classification of music emotion in China started late, but it has also made some achievements. Its research on music emotion classification is closely related to the development of music software functions. With the development of online music applications, music recommendation function has become an urgent demand [12]. Most of the single album and song list push services of various online music applications in the early stage were recommended based on a collaborative filtering algorithm. The biggest disadvantage of this method is that most of the recommended songs are current popular songs, which greatly reduces the recommendation probability of popular works [13, 14]. At the same time, the long-term recommendation of similar songs and song lists cannot meet people's demand for novelty [15]. The development of artificial intelligence and related technologies enables computers to analyze complex music emotions and automatically output emotion analysis results [16]. After feature extraction and selection of 37 music samples, some scholars improved the accuracy of feature classification through principal component analysis and linear discriminant analysis and effectively improved the accuracy of the emotion classifier based on k-NN [17]. Based on the relationship between music emotion and music genre, other scholars classify music emotion through SVM emotion classification and useful type information in music tags [18]. Other scholars have effectively extracted the emotional features in Chinese lyrics through the CNN pretraining word embedding model. The experimental results show that this method has higher accuracy than the traditional learning methods and other deep learning models [19]. Some scholars have constructed MIDI music emotion classification based on the BP neural network according to the characteristics of electronic music [20].

## 3. Construction of the Emotion Analysis Model of Electronic Music Based on PSO-BP Neural Network

Music is an artistic way for people to convey and express their emotions. The emotions in music can affect people's inner emotions, improve people's life beliefs, and show people's rich emotional world. At the same time, the emotional information contained in music has not only subjective initiative but also has overall fuzziness. Therefore, when analyzing data, the traditional logical reasoning method is difficult to deal with the emotion contained in it [21]. Based on the isomorphic correspondence between music acoustic vibration and human emotional activities described on the basis of psychology, this paper constructs the emotion recognition and analysis model of electronic music. Music emotion cognitive analysis model generally includes the music emotion psychological model and calculation model, that is, the data analysis model. Among the psychological models, Hevner model and Thayer model are commonly used models, which mainly discuss the characteristics of human emotion from the perspective of psychology [22]. Music emotion information is the basis of the electronic music emotion cognitive analysis model [23]. To some extent, people's psychological feeling process of music can be regarded as the process of music emotion information from acquisition, transformation, transmission, processing, and storage. Therefore, music [24], emotion information not only has subjectivity, objectivity, integrity, and fuzziness [25] but also has hierarchy. That is, people's cognition of electronic music emotion is hierarchical, as shown in Figure 1. The cognitive characteristics of different levels are one of the theoretical basis of the construction of electronic music emotion recognition and analysis model.

Different levels of cognitive characteristics are one of the theoretical bases for constructing the emotion recognition and analysis model of electronic music. In order to improve the accuracy of music emotion recognition, this paper proposes a music emotion recognition model based on different levels of features. Abandon the low-level features such as spectrum characteristics, chromaticity, and harmonic coefficient, and take the middle and high-level features closer to human cognition, including cognition, feeling, and memory, as the input of the emotion recognition model. The data set of music fragments is established, and the music emotion recognition is abstracted as a regression problem.

### 3.1. Emotional Feature Extraction of Electronic Music

Music emotion feature extraction is mainly from music lyrics, text information, and audio information. Emotion feature extraction in lyrics text is based on the sparse distribution of lyrics text, sentence length, repetition, emotion word recognition degree, and other characteristics [19]. As shown in formulas (1) and (2), it is the quantitative formula of a word recognition degree in electronic music:

(1) $$\begin{array}{c} \text{LMD}\left(w\right)=\sum_{i=1}^{K}\text{LMD}\left(w,i\right), \end{array}$$

(2) $$\begin{array}{c} \text{LMD}\left(w,i\right)=\frac{abs\left(P\left(w|i\right)-P\left(w|\neq i\right)\right)}{\sqrt{\text{max}\left(P\left(w|i\right),P\left(w|\neq i\right)\right)}}. \end{array}$$

The number of electronic music emotion classification is expressed as *K*, the probability of occurrence of word *w* in *i* emotion classification is expressed as *P*(*w|i*), and its probability of occurrence in *i* emotion classification accident category is expressed as *P*(*w|*≠*i*).

There are some differences in the energy of electronic music. The energy value of electronic music is higher, and its short-term energy calculation is shown in the following:

(3) $$\begin{array}{c} E_{m}=\sum_{N}^{N-1}{\left[y\left(n\right)\cdot c\left(n-m\right)\right]}^{2}. \end{array}$$

The electronic music signal is expressed as {*y*(*m*)}, its energy is expressed as *E*_*m*_, the window function is expressed as *c*(*m*), and the length of the electronic music signal frame is expressed as *N*.

The specific description of any frame of electronic music after smoothing through wavelet transform is shown in the following:

(4) $$\begin{array}{c} {\hat{Y}}_{t}\left(n\right)=\left\{{\hat{y}}_{t}\left(n,1\right),{\hat{y}}_{t}\left(n,2\right),\ldots ,{\hat{y}}_{t}\left(n,N\right)\right\}. \end{array}$$

Any frame of the processed electronic music is represented as ${\hat{Y}}_{t}\left(n\right)$. According to (4), the mean and variance of electronic music time domain can be calculated, as shown in the following:

(5) $$\begin{array}{c} E_{t}\left(n\right)=\frac{1}{N}\sum_{i=1}^{N}{\hat{y}}_{t}\left(n,i\right), \end{array}$$

(6) $$\begin{array}{c} D_{t}\left(n\right)=\frac{1}{N}\sum_{i=1}^{N}{\left[y_{t}\left(n,i\right)-E_{t}\left(n\right)\right]}^{2}, \end{array}$$

where the time-domain mean of electronic music is expressed as *E*_*t*_(*n*) and the variance is expressed as *D*_*t*_(*n*).

The expression of a frame of electronic music after wavelet transform smoothing in the frequency domain is shown in the following:

(7) $$\begin{array}{c} {\hat{Y}}_{f}\left(n\right)=\left\{{\hat{y}}_{f}\left(n,1\right),{\hat{y}}_{f}\left(n,2\right),\ldots ,{\hat{y}}_{f}\left(n,N\right)\right\}. \end{array}$$

A frame of electronic music processed in is expressed as ${\hat{Y}}_{f}\left(n\right)$, and the frequency domain mean and frequency domain variance of electronic music are calculated in combination with (7), as shown in the following:

(8) $$\begin{array}{c} E_{f}\left(n\right)=\frac{1}{N}\sum_{i=1}^{N}{\hat{y}}_{f}\left(n,i\right). \end{array}$$

(9) $$\begin{array}{c} D_{f}\left(n\right)=\frac{1}{N}\sum_{i=1}^{N}{\left[y_{f}\left(n,i\right)-E_{f}\left(n\right)\right]}^{2}, \end{array}$$

where the frequency domain mean of electronic music is expressed as *E*_*f*_(*n*) and the frequency domain variance is expressed as *D*_*f*_(*n*).

### 3.2. Emotion Model of Electronic Music Based on PSO-BP Neural Network

BP neural network is a multilayer feedforward neural network in the artificial neural network. It not only has the characteristics of adaptability, self-organization, and self-learning but also has the advantages of simple structure, mature algorithm, and accurate optimization. At the same time, its application in electronic music emotion recognition and analysis is more in line with the cognitive characteristics of human emotion in music recognition. However, with the increasing data related to emotional analysis and recognition of electronic music, the efficiency and accuracy of BP neural network decline [24]. In addition, BP neural network is easy to fall into a local minimum. Therefore, based on BP neural network, this paper introduces a particle swarm optimization algorithm to improve the efficiency and optimization ability of electronic music emotion analysis model.

BP neural network algorithm is also called error backpropagation algorithm. It is composed of three or more neural networks. The first layer is the input layer, the last layer is the output layer, the middle layer is the hidden layer, and the number of hidden layers is one or more layers. There is no connection between the nodes contained in each layer. Let the number of nodes in the input layer of the neural network be expressed as *d*, the number of nodes in the hidden layer is expressed as *m*, and the transfer function between nodes in each layer be sigmoid function, as shown in the following:

(10) $$\begin{array}{c} S\left(x\right)=\frac{1}{1+e^{-x}}, \end{array}$$

The output calculation formula of the neural network hidden layer is shown in the following:

(11) $$\begin{array}{c} D_{j}=S\left[\sum_{i=1}^{n}\left(R_{ij}x_{i}\right)\right]. \end{array}$$

Among them, *j*=1,2,…, *d*, the variable of the *i* input node is expressed as *x*_*i*_, and the excitation function of the hidden layer is expressed as *S*.

The output calculation formula of the output layer of the neural network is shown in the following:

(12) $$\begin{array}{c} O_{k}=S\left(\sum_{j=1}^{h}D_{j}R_{jk}\right). \end{array}$$

*k*=1,2,…, *m*.

Let the connection weight of the neuron between the input layer and the hidden layer of the BP neural network be expressed as *R*_*ij*_, and the connection weight of the neuron between the hidden layer and the output layer be expressed as *R*_*ik*_. The calculation formulas of the two are shown in the following:

(13) $$\begin{array}{c} R_{ij}\left(t+1\right)=R_{ij}\left(t\right)+\eta \left[\left(1-\theta \right)Q\left(t\right)+\theta Q\left(t-1\right)\right], \end{array}$$

(14) $$\begin{array}{c} R_{ik}\left(t+1\right)=R_{ik}\left(t\right)+\eta \left[\left(1-\beta \right)W\left(t\right)+\beta W\left(t-1\right)\right], \end{array}$$

where *i*=1,2,…, *n*;  *j*=1,2,…, *d*, *i*=1,2,…, *n*; *j*=1,2,…, *d*, the learning rate is expressed as *η* and *η* > 0, and the momentum factor is expressed as *θ* and 0 ≤ *θ* < 1, *Q*(*t*)=−*∂E*/*∂R*_*ij*_(*t*),  *W*(*t*)=−−*∂E*/*∂R*_*ik*_(*t*)..

PSO algorithm, namely particle swarm optimization algorithm, is an evolutionary computing technology derived from the study of bird predation behavior. It is a global optimization method based on swarm intelligence theory. PSO algorithm can not only optimize multidimensional space functions and dynamic objectives, but also has the advantages of fast convergence and good robustness.

Let the space of *L* dimension be the search space, and the number of particles contained in the population is *K*, then the position of the *j* particle in the population in the space can be expressed by *X*_*j*_=(*x*_*j*1_, *x*_*j*2_,…, *x*_*jl*_), and the optimal solution in the particle position is the global optimal individual, expressed as *P*_*j*_=(*p*_*j*1_, *p*_*j*2_,…, *p*_*jl*_), and the position velocity vector of the particle is expressed as *V*_*j*_=(*v*_*j*1_, *v*_*j*2_,…, *v*_*jl*_). As shown in (15) and (16), the position and velocity of each particle in the population after the iterative change:

(15) $$\begin{array}{c} v_{jl}\left(t+1\right)=g\cdot v_{jl}\left(t\right)+z_{1}\cdot r\;d\left(\right)\cdot \left(p_{jl}\left(t\right)-x_{jl}\left(t\right)\right)+z_{2}\cdot r\;d\cdot \left(p_{y}\left(t\right)-x_{jl}\left(t\right)\right), \end{array}$$

(16) $$\begin{array}{c} x_{jl}\left(t+1\right)=x_{jl}\left(t\right)+v_{jl}\left(t+1\right). \end{array}$$

In the formula, the inertia factor is expressed as *g*; the acceleration factor is expressed as *z*_1_, *z*_2_ and it is a normal number, *r*  *d* is a random value and *r*  *d* ∈ [0,1], and the current iterative algebra is expressed as *t*. Because the velocity and initial position of the particle swarm are generated randomly, the position and velocity of the particle swarm are iterated through (15) and (16). When both meet the termination conditions, the iteration of the particle swarm stops.

As shown in (17), it is the calculation formula of inertia weight in (15):

(17) $$\begin{array}{c} g=\left\{\begin{array}{c} g_{\max}-\frac{\left(g_{\max}-g_{\min}\right)\left(s-s_{\text{ave}}\right)}{s_{\max}-s_{\text{ave}}},\;s\geq s_{\text{ave}},\\ g_{\max},\;s<s_{\text{ave}}. \end{array}\right.. \end{array}$$

The fitness value of particles is expressed as *s*, the average fitness value of particles is expressed as *s*_ave_, and the largest fitness value in particle swarm is expressed as *s*_max_.

Figure 2 shows the flow chart of PSO Algorithm Optimizing BP neural network.

As can be seen from Figure 2, optimizing the weight and threshold of the BP neural network through the PSO algorithm needs to recover the parameters such as particle number, position, and learning factor contained in the PSO algorithm. Then BP neural network is constructed according to the number of input and output signals, and its weight and threshold length are initialized. Then they are encoded to obtain the initial population of the PSO algorithm.

The BP neural network is optimized by the PSO algorithm, and then the optimization iteration is carried out. The extreme values of particles and particle swarm are determined by the fitness values of each group of particles, in which the best position is the best position in the history of particles in the optimization iteration process. The iterative update of particle speed and position is carried out according to the formula. When the fitness reaches the expected accuracy or the maximum number of iterations is completed, the optimization iteration stops, and the current position of the particle is the optimal solution to solve the target. The optimal weight and threshold of the BP neural network are obtained by decoding. If the conditions are not met, the optimization iteration will be carried out again.

## 4. Application Experiment of the Emotion Analysis Model of Electronic Music Based on PSO-BP Neural Network

This study collects 190 electronic music samples, of which 50 electronic music are randomly selected as the test sample set, and 140 electronic music are the training set of the model. The emotion of electronic music is mainly divided into eight types according to the Hevner model, including cheerful, lyrical, calm, quiet, sad, passionate, resolute, and angry emotion. The output performance of the BP neural network is greatly affected by the number of hidden layer nodes in its structure. Before the emotional analysis of electronic music, it is necessary to determine the optimal number of nodes of the BP neural network through training. Let the number of iterations of node training be 20, as shown in Figure 3, which is the relationship between the number of hidden layer nodes of the BP neural network and the error rate of BP neural network training results. It can be seen from the results in the figure that the increase of nodes in the hidden layer in the BP neural network structure will continuously improve the accuracy of its training results. When the number of hidden layer nodes is less than 100, the error rate will be greatly reduced with the increase of the number of nodes. When the number of hidden layer nodes exceeds 100, the error rate decreases gradually with the increase of the number of nodes. At the same time, from the perspective of time cost, the excessive number of hidden layer nodes contained in the BP neural network will have a great impact on its operation efficiency. Therefore, considering all factors and influences, the number of hidden layer nodes in BP neural network is 100.

The maximum number of iterations of the emotion analysis model of electronic music based on the PSO-BP neural network is 1500.  Figure 4 shows the comparison of the optimal individual fitness values of the PSO-BP neural network and BP neural network.

As can be seen from Figure 4, the BP neural network needs 65 iterations to achieve the convergence effect, and there are short-term fluctuations after convergence. The PSO-BP neural network can converge after 46 times, and the convergent curve tends to be stable. This shows that compared with BP neural network, PSO-BP neural network has a faster convergence speed, more stable operation, and better performance.

As shown in Figure 5, the accuracy of pos-bp neural network and traditional BP neural network in the emotional classification of electronic music text is compared. Thirty-two pieces of electronic music were randomly selected from the test sample set and divided into four groups for the text emotion classification test. On the whole, the classification accuracy of the PSO-BP neural network is higher than that of the traditional BP neural network. When the traditional BP neural network classifies the emotion of four groups of electronic music, the accuracy fluctuates greatly. The accuracy of emotion classification of four groups of electronic music by PSO-BP neural network has been maintained at a stable level, and its operation is more stable.

Figure 6 shows the emotional analysis results of electronic music in the test sample set based on PSO-BP neural network electronic music emotional analysis model. It can be seen from the results in the figure that based on the PSO-BP neural network electronic music emotion analysis model, the data analysis is carried out from the characteristics of electronic music and the pitch, length, speed, strength, and timbre of its notes. On the basis of the data analysis results, the emotion analysis of electronic music is further carried out and the corresponding emotion analysis results are output.

As shown in Figure 7, it is the comparison between the emotional analysis results of electronic music based on the PSO-BP neural network emotional analysis model and the actual results. It can be seen from the results in the figure that the error between the electronic music emotion analysis results obtained by the electronic music emotion analysis model based on PSO-BP neural network and the actual results is small, which shows that it has a high accuracy of electronic music emotion analysis and meets the expected requirements.

To sum up, compared with the traditional BP neural network, PSO-BP neural network has a faster convergence speed, avoids the problem that BP neural network is easy to fall into local optimization, and provides a more stable operation performance for later model training and testing. Multiple neural networks can be initialized by different parameter values, and the smallest one can be taken as the result. Just like enterprise job rotation, try to start from different positions, which can avoid falling into the trap of thinking that the current position is the most suitable. In addition, “simulated annealing” technology can be used. Simulated annealing will accept worse results than the current with a certain probability at each step, which helps to “jump out” of the local minimum. As time goes by, the probability of “optimal solution” should be continuously reduced. The emotion analysis model of electronic music based on the PSO-BP neural network can complete the emotion analysis of electronic music lyrics and music melody with high accuracy. There is less error between the analysis results and the actual results, which meets the expected requirements of the model.

## 5. Conclusion

With the development of electronic music, the type and quantity of electronic music are increasing. People need to spend a lot of time and energy choosing their preferred type in a large number of electronic music. Therefore, the classification of electronic music and the research of the emotion analysis model have become the research focus of electronic music operation. However, the previous emotion analysis models of electronic music have large errors in emotion recognition in electronic music, which cannot meet people's more and more detailed needs. The development of artificial intelligence and data analysis technology provides a new development direction for electronic music emotion analysis. Therefore, this paper proposes electronic music emotion analysis based on PSO-BP neural network and data analysis. Based on the BP neural network optimized by the PSO algorithm and combined with the extraction of emotional features of electronic music, the emotion of electronic music is recognized and analyzed. The experimental results show that compared with BP neural network, PSO-BP neural network has a faster convergence speed and better optimal individual fitness value, avoids falling into local optimal solution and provides a more stable running state for its training and testing. At the same time, *p* the BP neural network optimized by PSO has a lower error rate in the emotional analysis of electronic music lyrics, which can better identify and classify emotions. According to the characteristics of electronic music, PSO-BP neural network can effectively identify and analyze the emotion of electronic music with high accuracy, which is close to the actual situation and meets the expected requirements. In this paper, the emotion analysis model of electronic music based on the PSO-BP neural network still has many shortcomings, which need to be further improved and improved to improve the performance of the emotion analysis model of electronic music. Later, it needs to be further refined according to the characteristics of electronic music, which is closer to the needs of human emotion.

## Figures and Tables

**Figure 1:** Cognitive level characteristics of electronic music emotion.

**Figure 2:** Flow chart of PSO Algorithm Optimizing BP neural network.

**Figure 3:** The relationship between the number of hidden layer nodes of the BP neural network and the error rate of BP neural network training results.

**Figure 4:** Comparison of optimal individual fitness between PSO-BP neural network and BP neural network.

**Figure 5:** Comparison results of PSO-BP neural network and traditional BP neural network in emotion classification accuracy of electronic music.

**Figure 6:** The emotion analysis results of electronic music in the test sample set are analyzed based on PSO-BP neural network emotion analysis model of electronic music.

**Figure 7:** Comparison between the emotional analysis results of electronic music and the actual results based on the PSO-BP neural network emotional analysis model of electronic music.

## Data Availability

The data used to support the findings of this study are available from the corresponding author upon request.
